# Establishment of a Risk Prediction Model for Pulmonary Infection in Patients with Advanced Cancer

**DOI:** 10.1155/2022/6149884

**Published:** 2022-05-30

**Authors:** Liangliang Yang, Xiaolong Xu, Qingquan Liu

**Affiliations:** ^1^School of Clinical Medicine, Beijing University of Chinese Medicine, Beijing 100029, China; ^2^Department of Critical Care Medicine, Beijing Hospital of Traditional Chinese Medicine, Capital Medical University, Beijing 100010, China

## Abstract

**Objective:**

Based on clinical data, the risk prediction model of pulmonary infection in patients with advanced cancer was established to predict the risk of pulmonary infection in patients with advanced cancer, and intervention measures were given in advance.

**Methods:**

The clinical data of 2755 patients were divided into infection group and control group according to whether they were complicated with lung infection. 1609 patients' data from January 2016 to December 2018 served as the training set, and 1166 patients' data from January 2019 to December 2020 served as the testing set. Demographics, whether the primary cancer was lung cancer, lung metastasis, the pathological classification of lung cancer patients, the number of metastases, history of surgery, history of chemotherapy, history of radiotherapy, history of central venous catheterization, history of hypertension, diabetes, and whether with myelosuppression were recorded. The presence of concurrent pulmonary infection was recorded and defined as the primary outcome variable. Stepwise forward algorithms were applied to informative predictors based on Akaike's information criterion. Multivariable logistic regression analysis was used to develop the nomogram. An independent testing dataset was used to validate the nomogram. Receiver-operating characteristic curves and the Hosmer-Lemeshow test were used to assess model performance.

**Results:**

The sample included 2755 patients with advanced cancer. An independently validated dataset included 1166 patients with advanced cancer. In the training dataset, gender, age, lung cancer as primary cancer, the pathological classification of lung cancer patients, history of chemotherapy, history of radiation therapy, history of surgery, the number of metastases, presence of central venous catheterization, and myelosuppression were identified as predictors and assembled into the nomogram. The area under curve demonstrated adequate discrimination in the validation dataset (0.77; 95% confidence interval, 0.74 to 0.79). The nomogram was well calibrated, with a Hosmer-Lemeshow *χ*^2^ statistic of 12.4 (*P* = 0.26) in the testing dataset.

**Conclusions:**

The present study has proposed an effective nomogram with potential application in facilitating the individualized prediction of risk of pulmonary infection in patients with advanced cancer.

## 1. Introduction

With the deterioration of the ecological environment, the aging of the population, and a series of other problems, the incidence of malignant tumors is increasing. Cancer has become the second leading cause of death in the world after cardiovascular and cerebrovascular diseases, bringing a huge economic burden to the public health system [1]. Patients with malignant tumors are at high risk of serious infection [2]. Infection in cancer patients may delay the initiation of chemotherapy and reduce the dose that can be administered. In addition, it significantly lengthens hospital stays, increases the cost of treatment, and increases morbidity and mortality [3]. Due to the consumption of the disease itself and long-term, repeated chemotherapy, radiotherapy, and other factors, patients with advanced cancer have low immunity and are prone to various infections, especially pulmonary infections, which occupy the primary position in various systemic infectious diseases [4, 5]. In a retrospective study of 102 advanced cancer patients in Australia, the overall infection rate was 36.3%, and in this study, lung infections (22.9%) were the third highest after urinary tract infections (42.5%) [6]. The occurrence of infection will seriously affect the comprehensive treatment of patients with advanced cancer and reduce the quality of life of patients, and a considerable number of patients with advanced cancer eventually die of lung infection. Thus, early identification and aggressive treatment of infection is critical for overall survival of cancer patients, and delayed administration of appropriate anti-infective therapy is associated with poorer prognosis [7].

Most of the existing prediction models are models to predict the survival rate and prognosis of patients with advanced cancer [8], but there is no model to predict the risk of pulmonary infection in patients with advanced cancer. We established the prediction model for the risk of pulmonary infection in patients with advanced cancer to help clinicians individually predict the risk of disease, so as to carry out prevention and treatment. Nomograms have been considered an effective visualization tool for individual predictions from multivariable models [9]. The purpose of the present study was to develop and validate a nomogram for the clinical prediction of the severity of postoperative symptoms using an independent dataset for clinical prediction of pulmonary infection risk in patients with advanced cancer.

## 2. Materials and Methods

### 2.1. The Research Object

The study samples were collected from stage IV malignant tumor patients admitted to the Affiliated Tumor Hospital of Xinjiang Medical University from January 2016 to December 2020. This study was approved by the Medical Ethics Committee of the Affiliated Tumor Hospital of Xinjiang Medical University (2020BL02-064-03).

Inclusion criteria: patients with stage IV malignant tumor: ① patients with malignant tumor clearly diagnosed by pathology or cytology; ② there is distant metastasis (the tumor spreads to other parts of the body). Pulmonary infection: X-ray examination of new or advanced pulmonary infiltration shadow plus two or more of the following clinical symptoms: ① fever over 38°C, ② leukocyte increase or decrease, ③ and discharge from purulent air duct. Patients younger than 10 years and older than 90 years were excluded.

### 2.2. Study Variables

The clinical data of the two groups were read in detail one by one, and relevant information was collected and summarized by retrospective study, including gender, age, ethnicity, whether the primary cancer is lung cancer, the pathological classification of lung cancer patients, whether there is lung metastasis, the number of metastases, whether there is a history of surgery, whether there is a history of chemotherapy, whether there is a history of radiotherapy, whether there is a history of central vein catheterization, whether there is hypertension, whether there is diabetes, and whether there is bone marrow suppression.

We defined, integrated, and grouped the variables in the data: (1) patients were divided into surgical group and nonsurgical group according to whether they had received surgical treatment; (2) according to the situation of patients receiving radiotherapy, patients were divided into radiotherapy group and nonradiotherapy group; (3) patients were divided into chemotherapy group and nonchemotherapy group according to their chemotherapy; (4) patients were divided into myelosuppression group and nonmyelosuppression group according to the status of myelosuppression; (5) according to whether the patients have diabetes, the patients are divided into diabetic group and nondiabetic group; (6) patients were divided into hypertensive group and nonhypertensive group according to whether they had hypertension or not; (7) patients were divided into lung cancer group and nonlung cancer group according to whether the primary cancer was lung cancer; (8) the pathological types of lung cancer patients are divided into adenocarcinoma, squamous cell carcinoma, small cell carcinoma, sarcomatoid carcinoma, neuroendocrine carcinoma, and choriocarcinoma; (9) patients were divided into pulmonary metastasis group and nonpulmonary metastasis group according to whether the distant metastasis site was pulmonary metastasis; (10) the patients were divided into Han, Uygur, Kazak, Hui, and other ethnic groups according to their ethnic groups; (11) patients were divided into central vein catheterization group and noncentral vein catheterization group according to whether there was central vein catheterization. The main outcome of this study was whether there was pulmonary infection.

1609 patients' data from January 2016 to December 2018 served as the training set, and 1166 patients' data from January 2019 to December 2020 served as the testing set, which were used to establish training datasets and validation datasets, respectively. The training dataset included 664 patients in the infection group and 945 patients in the control group, and the validation dataset included 483 patients in the infection group and 683 patients in the control group. The training dataset was used to develop the prediction model and nomogram, and the testing dataset was used to evaluate its predictive performance.

### 2.3. Sample Size

Our sample size calculation was determined by our primary objective (binary outcome). In prediction studies (e.g., those used for nomogram development and validation), the number of outcome events will dictate the effective sample size. On the basis of some empirical investigations, the sample was defined to have at least 10 outcome events per variable (EPV) or, more precisely, per estimated parameter [10, 11].

Our sample and the number of events exceeded that found using the EPV approach for determining sample sizes and can, therefore, be expected to provide robust estimates.

### 2.4. Statistical Analysis

Using EXCEL spreadsheets manages the collected data and then transferred to STATA, version 15.0, for Windows (StataCorp, College Station, TX) for statistical analysis. The training dataset was used to develop the prediction model in the final logistic regression. A bivariate analysis was performed using the Mann–Whitney *U* test for continuous variables and the Fisher exact c2 test for categorical variables, with “whether pulmonary infection” as the outcome. Variables for inclusion in the final logistic regression model were carefully chosen using forward stepwise selection, with Akaike's information criterion (AIC) as the stopping rule [12, 13]. The AIC value for the final model was minimized with the smallest number of variables. Using the Nomolog feature in STATA version 15.0 derives a rote plot from the results of multivariate logic analysis. We subsequently validated the prediction model by examining both nomogram discrimination and calibration using the testing dataset.

The rotors constructed from the training dataset were also used to calculate the probability of pulmonary infection outcomes in the validated dataset. To assess model discrimination, we calculated the area under the receiver-operating characteristic (ROC) curve. The calibration curve was evaluated using the Hosmer-Lemeshow goodness of fit test and the validation sample. All statistical tests were 2-sided, and *P* values of <0.05 were considered statistically significant.

## 3. Results

1609 patients' data from January 2016 to December 2018 were used to establish the rosette prediction model, and 1166 patients' data from January 2019 to December 2020 were used to evaluate its performance.

The training dataset included 664 patients in the infected group and 945 patients in the control group. Among them, there were 932 males and 677 females, 621 patients with lung cancer, 300 patients with pulmonary metastasis, 707 patients with a history of surgery, 1344 patients with a history of chemotherapy, 147 patients with a history of radiotherapy, 111 patients with central venous catheters, 21 patients with bone marrow suppression, 106 patients with hypertension, 50 patients with diabetes, and 771 patients with only one metastasis. 442 had 2 metastases, 256 had 3 metastases, 108 had 4 metastases, 22 had 5 metastases, and 1 had 6 metastases. Among patients with lung cancer, 489 had adenocarcinoma, 62 had squamous cell carcinoma, 64 had small cell carcinoma, 7 had sarcomatoid carcinoma, 5 had neuroendocrine carcinoma, and 1 had chorionic carcinoma. The bivariate relationship between the predictive variables of the training dataset and concurrent pulmonary infection is shown in Table 1.

After using the multivariate regression model for variable selection, choose the gender, age, whether primary cancer for lung cancer, with lung metastasis lesions, the pathological classification of lung cancer patients, the number of metastases, with or without history of chemotherapy, with or without radiotherapy, with or without history of surgery, central venous catheter or not, and whether have myelosuppression as a complicated with lung infection probability; the best predictor of the subset are shown in Table 2. The nomogram that incorporated these predictors is presented in Figure 1. In the picture, “Hyper” stands for hypertension, 0 for no hypertension, and 1 for hypertension. “Race” represents ethnic groups. One is Han, two is Uygur, three is Kazak, four is Hui, and five is other ethnic groups. Gender: 1 is male, 2 is female. “Meta” represents the number of metastases. “Pathology” represents the pathological classification of lung cancer patients, 1 represents adenocarcinoma, 2 represents squamous cell carcinoma, 3 represents small cell carcinoma, 4 represents sarcomatoid carcinoma, 5 represents neuroendocrine carcinoma, and 6 represents choriocarcinoma, “Veni” represents with or without central vein catheterization, 0 represents without central vein catheterization, and 1 represents with central vein catheterization. “Radio” represents history of radiotherapy, 0 represents no history of radiotherapy, and 1 represents history of radiotherapy. “Primary” indicates whether the primary cancer is lung cancer, 0 indicates that the primary cancer is not lung cancer, and 1 indicates that the primary cancer is lung cancer. “Chemo” represents history of chemotherapy, 0 represents no history of chemotherapy, and 1 represents history of chemotherapy; “myelo” represents myelosuppression, 0 represents without myelosuppression, 1 represents with myelosuppression, “oper” represents surgical history, 0 represents no surgical history, and 1 represents surgical history.

The nomogram had good discriminative power with an area under the ROC curve of 0.77 (95% confidence interval, 0.74 to 0.79) and 0.77 (95% confidence interval, 0.75 to 0.80) in the training and testing datasets, respectively (Figures 2(a) and 2(b)). In addition, the nomogram was well calibrated with a Hosmer-Lemeshow *χ*^2^ statistic of 12.4 (*P* = 0.26) and 8.3 (*P* = 0.59) in the training and testing datasets, respectively (Figure 3).

Furthermore, the decision curve analysis for the nomogram is presented in Figure 4. We did DCA on our prediction model to assess the net benefit that patients could receive. As the decision curve indicates, the nomogram model has an obvious net benefit for almost all threshold probabilities, especially in threshold probabilities of 18%-90%. However, if the threshold probability were less than 10%, the net benefit of nomogram was equivalent to predicting positive results for all patients.

## 4. Discussion

Our study has developed and assessed a nomogram for predicting the risk of lung infection in patients with advanced cancer. It is well calibrated and discriminated for the individualized prediction and facilitates individual treatment. This will improve clinical decision-making for clinicians and patients to get more net benefits.

Our results show that the primary cancer, lung cancer, is a risk factor for pulmonary infection in patients with advanced cancer. According to relevant epidemiological studies, lung infection is the complication with the highest incidence of lung cancer patients after surgery, radiotherapy, and chemotherapy [14]. This may be related to bronchial obstruction, immunosuppression, bone marrow suppression, the destruction of local defense function caused by tumor invasion, and the destruction of tumor and normal tissue [15]. Previous studies have also shown that the most common type of infection in lung cancer patients is lung infection [16]. Age is closely related to the incidence of advanced cancer patients complicated with lung infection, which may be related to elderly patients with the body function and decline in immune function, increased with age, body function of various organs gradually degraded, respiratory function, structure, and so on; a series of degeneration, elasticity, and vital capacity of lung tissue also gradually reduced the respiratory tract mucosa atrophy. The decrease of the ability of the epithelial cilium system, the decrease of the lung defense and protection function, the degeneration of the clearance function of the mucosal cilium system, the decrease of specific immune function, and the decrease of the reactivity to disease lead to the increase of susceptibility to infectious diseases [17]. Research by Miura et al. confirms this view [18]. However, unlike previous studies, our results suggest that no prior radiotherapy or chemotherapy is a risk factor for pulmonary infection in patients with advanced cancer. There are two possible explanations for this result. One is patient selection bias. Almost all advanced cancer patients who receive chemotherapy and radiation are relatively young and need to be in good enough physical functioning to tolerate these destructive treatments. The second is to help patients control the development of cancer disease through chemotherapy and radiotherapy treatment, improve the nutritional status of patients with advanced cancer, and improve the quality of life of patients. Studies have found that although chemotherapy inhibits the immune system to a certain extent, it also has a positive regulation effect on the immune system, which can enhance the immune function and enhance the antitumor effect, which can be regarded as a richer pharmacological effect besides the cytotoxicity of chemotherapy drugs. Chemotherapy to activate the immune mechanism is mainly divided into two parts: effects on tumor “indirect activation” and “activated directly” effects on immune cells, as a kind of indirect immune activation and chemotherapy in the process to improve the previous state of immune tolerance and to induce the immune function and activation of antitumor immune to remove lesions [19]. Tumor radiation therapy can affect the body's immune function; the latest research shows that the appropriate radiation therapy can be regulated by the tumor microenvironment, activate the body's immune cells, and release the death danger signals and, in turn, activate the immune response and generate a bystander or far effect; the bystander effect refers to the local after radiotherapy can cause systemic reactions, thus promoting tumor regression in distant nonradiotherapy areas [20]. In our results, men with advanced cancer were more likely to develop lung infections than women, which may be due to the fact that more men than women smoke. About 37 percent of adult men worldwide smoke, according to statistical studies [21]. In 2002, among people aged 15 and over, the active smoking rate was 66.0 percent for males and 3.1 percent for females [22]. In China, the smoking rate of men aged 15 and above is as high as 52.1%, and that of women is 2.7%. The number of men smoking is significantly higher than that of women [23]. After the harmful substances produced by tobacco burning enter the body, the first damage is the respiratory system, causing damage to the mucous membrane of the respiratory tract, the release of chemotactic inflammatory cells and inflammatory factors, and then trigger immune inflammatory response [24]. Studies have shown that compared with nonsmokers, smokers with lower respiratory tract infection and health examination can increase Il-4 and IL-5 in induced sputum and decrease INF-*γ*, and increased smoking index can inhibit the expression of INF-*γ*, imbalance of TH1/TH2 system, and disorder of internal immune defense mechanism, affecting the normal immune response after infection [25]. Central venous catheterization (CVC) is a catheter placed in a large vein (such as the internal jugular vein, subclavian vein, or femoral vein) and is often used for chemotherapy or total parenteral nutrition [26]. Central venous catheters provide safe vascular access for critically ill and chronically ill patients [27]. Patients with cancer often require treatment and parenteral nutrition using central catheters and are at high risk for central catheter-related infections [28]. Infection is the most common complication of CVC use [29]. Central venous catheter infections occur in 2-43% of patients with CVC [30]. Myelosuppression occurs in some patients during chemotherapy, which leads to a decrease in the number of granulocytes [31]. Granulocytes, the main component of blood white blood cells, play an important role in host defense during tissue injury, inflammation, and infection through their ability to migrate, phagocytose, and produce reactive oxygen species [32, 33]. The reduction of immunity and defense function caused by bone marrow suppression is malignant important factor of secondary infection in tumor patients [34]. The more serious the bone marrow suppression, neutrophils lack for a long time, will increase the pathogenic bacteria invasion mechanism, leading to a large number of pathogenic microorganisms in the body and then reduce the immune function of the body [35]. Surgical history is a risk factor for pulmonary infection in patients with advanced cancer. Experimental and clinical studies have shown that surgical trauma significantly affects the immune system, including specific and nonspecific immune responses. No matter what type of surgery, it triggers a systemic immune response [36]. Major surgery has been shown to lead to postoperative immunosuppression. Specifically, open surgery results in (1) decreased chemotaxis of lymphocytes and neutrophils, (2) decreased activity of natural killer cells, (3) decreased lymphocyte and macrophage interactions, and (4) decreased delayed hypersensitivity (DTH) [37]. Many experimental and clinical studies have shown that surgical trauma reduces neutrophil functions such as chemotaxis, superoxide, and leukotriene-C4 production [38]. Tissue damage after surgery and trauma leads to a decrease in cell-mediated immunity, which increases the risk of infection [39].

The nomogram is a tool that can graphically display the results of a regression model. It involves drawing a cluster of line segments, by which it is possible to easily calculate the risk for different individuals [40]. We developed a graph predicting pulmonary infection in patients with advanced cancer and combined it with predictors. The nomogram is a valuable innovation that can be used to individualize the prediction of disease risk, leading to individualized prevention and treatment. Its use can improve clinical decision-making for clinicians and patients, resulting in greater net benefit. The nomogram can help users obtain the probability of lung infection in patients with advanced cancer. Accurate prediction of pulmonary infection in patients with advanced cancer is helpful to improve the therapeutic effect of patients. Once it is confirmed that some patients are prone to pulmonary infection, high attention should be paid to it in clinical work, and intervention measures should be implemented.

The current study still has some limitations. First, it was a retrospective study with a relatively small sample size. Secondly, the samples were all from single centers, with regional bias. This study examined only a small subset of the entire patient population, so the reproducibility, generality, and applicability of our findings to other populations are unclear, and these findings need to be validated in future intervention studies. Third, if multicenter prospective external validation is used, the prediction performance of the rosette map will be better, and the generalization of the rosette map should be verified in multicenter studies with large sample sizes. However, this study used 10 factors to establish a graph of the risk of pulmonary infection in patients with advanced cancer. It can be easily used to individually predict the risk of pulmonary infection in patients with advanced cancer. Despite its limitations, it is hoped that the graph will provide a convenient and useful tool for prediction and patient counseling.

## Figures and Tables

**Figure 1:** Nomogram to estimate the likelihood of developing lung infections in patients with advanced cancer. Find the predictor points on the uppermost point scale that correspond to each patient variable and total them. The total score projected on the bottom scale indicates the percentage of probabilities of concurrent pulmonary infection.

**Figure 2:** Receiver-operating characteristic (ROC) curves of the nomograms in the training (a) and testing (b) datasets. The nomogram had good discriminative power with an area under the ROC curve of 0.77 (95% confidence interval, 0.74 to 0.79) and 0.77 (95% confidence interval, 0.75 to 0.80) in the training and testing datasets, respectively. The discrimination is quantified by calculating the area under the ROC curve (AUC). An AUC of 0.5 indicates no discrimination, and an AUC of 1.0 represents excellent discrimination.

**Figure 3:** The calibration curve of nomogram for predicting developing pulmonary infection in the training ((a) *P* = 0.26) and testing ((b) *P* = 0.59) dataset. The calibration focused on the accuracy of the absolute risk prediction of the model (i.e., the consistency between the probability of serious postoperative severity predicted by the model and that actually observed). The *y*-axis represents the actual rate of developing pulmonary infection. The *x*-axis represents the predicted probability of developing pulmonary infection. For a nomogram with better calibration, the scatter points should be arranged along a 45° diagonal line. The Hosmer-Lemeshow goodness-of-fit test is often used to compare whether significant differences exist between the prediction probability and the actual occurrence, with *P* > 0.05 indicating no statistically significant difference, and the calibration of the model was good.

**Figure 4:** Decision curve analysis for the nomogram. The *y*-axis measures the net benefit. The blue line represents the nomogram. The green line represents the assumption that all patients have extended operation time. The pink line represents the assumption that no patients have extended operation time. The decision curve showed that if the threshold probability of a patient or doctor is >18%, using the nomogram in the current study to predict extended operation time adds more benefit than the treat-all-patients scheme or the treat-none scheme.

**Table 1:** The training dataset predicted a bivariate relationship between variables and concurrent pulmonary infection.

Study variable	Control group	Infection group	*P* value
*N*	945	664	
Gender			<0.01
Male	501 (53.0%)	431 (64.9%)	
Female	444 (47.0%)	233 (35.1%)	
Age, median (IQR)	57.0 (48.0, 67.0)	63.0 (54.0, 73.0)	<0.01
Lung metastases			<0.01
No	791 (83.7%)	518 (78.0%)	
Yes	154 (16.3%)	146 (22.0%)	
Pathology			<0.01
Other cancers	706 (74.7%)	278 (41.9%)	
Adenocarcinoma	203 (21.5%)	286 (43.1%)	
Squamous cell carcinomas	14 (1.5%)	48 (7.2%)	
Small cell lung cancer	21 (2.2%)	43 (6.5%)	
Sarcomatoid carcinoma	1 (0.1%)	6 (0.9%)	
Neuroendocrine carcinoma	0 (0.0%)	2 (0.3%)	
Choriocarcinoma	0 (0.0%)	1 (0.2%)	
Race			<0.01
The Han nationality	641 (67.8%)	506 (76.2%)	
Uighurs	192 (20.3%)	94 (14.2%)	
Kazak	52 (5.5%)	20 (3.0%)	
The hui nationality	36 (3.8%)	31 (4.7%)	
Other ethnic groups	24 (2.5%)	13 (2.0%)	
Whether the primary cancer is lung cancer			<0.01
No	706 (74.7%)	282 (42.5%)	
Yes	239 (25.3%)	382 (57.5%)	
History of surgery			0.36
No	539 (57.0%)	363 (54.7%)	
Yes	406 (43.0%)	301 (45.3%)	
History of chemotherapy			<0.01
No	103 (10.9%)	162 (24.4%)	
Yes	842 (89.1%)	502 (75.6%)	
History of radiation therapy			0.14
No	850 (89.9%)	612 (92.2%)	
Yes	95 (10.1%)	52 (7.8%)	
Diabetes			0.38
No	919 (97.2%)	640 (96.4%)	
Yes	26 (2.8%)	24 (3.6%)	
Hypertension			0.41
No	887 (93.9%)	616 (92.8%)	
Yes	58 (6.1%)	48 (7.2%)	
Bone marrow suppression			0.18
No	936 (99.0%)	652 (98.2%)	
Yes	9 (1.0%)	12 (1.8%)	
Central vein catheterization			<0.01
No	899 (95.1%)	599 (90.2%)	
Yes	46 (4.9%)	65 (9.8%)	
Number of metastases, median (IQR)	2.0 (1.0, 3.0)	1.0 (1.0, 2.0)	0.02

**Table 2:** Predictors of pulmonary infection in patients with advanced cancer in the final regression model of the training dataset.

Related factors	*β*	OR	95% CI	*P* value
History of chemotherapy	-2.003	0.135	-2.398–-1.609	≤0.001
Whether the primary cancer is lung cancer	0.925	2.524	0.534-1.317	≤0.001
History of radiation therapy	-1.564	0.209	-2.076–-1.052	≤0.001
Central vein catheterization	0.792	2.208	0.326-1.258	≤0.001
Pathology	0.403	1.497	0.156-0.650	≤0.001
Gender	-.276	0.759	-0.510–-0.041	0.021
Age	0.244	1.025	0.015-0.338	≤0.001
Bone marrow suppression	1.346	3.842	0.347-2.343	0.008
History of surgery	0.228	1.256	-0.014-0.470	0.065
Number of metastases	-0.113	0 .893	-0.227-0.001	0.052
Constant	-.186	0.830	-1.018-0.646	0.662

## Data Availability

The data used to support the findings of this study are available from the corresponding author upon request.
